# Anticonvulsant Activity of *trans*-Anethole in Mice

**DOI:** 10.1155/2022/9902905

**Published:** 2022-05-14

**Authors:** Erika da Guedes, Leandro Rodrigo Ribeiro, César Alves Carneiro, Aline Matilde Ferreira Santos, Álefe Brito Monteiro, Humberto Hugo Nunes de Andrade, Ricardo Dias Castro, Flávio Freitas Barbosa, José Maria Barbosa Filho, Reinaldo Nóbrega de Almeida, Mirian Graciela Stiebbe Salvadori

**Affiliations:** ^1^Health Sciences Center/Federal University of Paraíba, Brazil; ^2^Department of Odontology/Federal University of Paraíba, Brazil; ^3^Department of Psychology/Federal University of Paraíba, Brazil; ^4^Department of Pharmaceutical Sciences/Federal University of Paraíba, Brazil; ^5^Department of Physiology and Pathology/Federal University of Paraíba, Brazil

## Abstract

Epilepsy is a chronic neurological disorder affecting 1-2% of world population, and one-third of patients are refractory to pharmacological treatment. This fact has stimulated research for new antiepileptic drugs and natural products have been an important source. *trans*-Anethole (TAN) is a phenylpropanoid, component of some essential oils, extracted from plants, and its effects have been little studied. Therefore, this study is aimed at investigating the TAN effect in classic seizure models and evaluate the electroencephalographic (EEG) profile of animals treated with this substance. For this, Swiss male mice (*Mus musculus*) were used, and the lethal dose was evaluated and subsequently submitted to the test maximal electroshock (MES), the pentylenetetrazole- (PTZ) induced seizure test, and the EEG profile. Initially, the LD50 for TAN was estimated in 1000 mg/kg (i.p.) dose and there was no sign of acute toxicity or death. In the MES test, TAN 300, i.p. (12.00 ± 2.9 s) and 400 mg/kg, i.p. (9.00 ± 4.4 s) doses was able to decrease tonic seizures duration induced by electric discharge (0.5 mA, 150 pulses/s, for 0.5 s). In the PTZ test (75 mg/kg, i.p.), TAN 400 mg/kg, i.p. increased the latency to myoclonic jerks (80.0 (56.0–134.0)), the latency totonic-clonic seizures (900.0 (861.0–900.0) and decrease seizure duration (0.0 (0.0–10.0)). No deaths were found in this groups compared to vehicle. EEG analysis showed an amplitude decrease of waves (ratio of baseline) in TAN 300 (1.82 ± 0.23) and 400 mg/kg (1.06 ± 0.16) groups. In this way, TAN at 400 mg/kg was able to inhibit and/or attenuate seizures by increasing the time for the onset of spasms and convulsions, as reducing the duration of seizures. The EEG profile corroborate with this results showing a reduction in the amplitude of waves compared to the PTZ group. Thus, TAN showed an anticonvulsant effect in all experimental models performed, behavioral and electroencephalographic.

## 1. Introduction

Epilepsy is a chronic neurological disease characterized by spontaneous recurrent seizures, through transitory signs due to abnormal, excessive, or synchronous brain neuronal activity [1, 2]. Seizure episodes are results of neurons excessive electrical discharges due to disrupted balance between excitation and inhibition in the brain. These mechanisms are associated with a complex neurotransmitter process involving glutamatergic, cholinergic, and GABAergic systems [3, 4].

Although the pathophysiology of seizure is not well defined, a generally accepted principle is that glutamate, as the major excitatory neurotransmitter, is excessively released and binds to its receptors, especially to NMDA and AMPA, triggering seizures. On the other hand, inhibition of this pathway occurs through the release of gamma-aminobutyric acid (GABA) by inhibitory interneurons. In this way, drugs that inhibit glutamate receptors or enhance GABA function are able to prevent seizures [5, 6].

Despite the access to a vast pharmacological resource, many patients still have seizures and nearly 30% of them are considerate drug therapy resistant, without adequate response to treatment. Besides, current clinical antiepileptic drugs have many side effects [7].

In traditional medicine, some of the plants used for epilepsy treatment have been scientifically shown to possess promising activity in animal models used in the screening of antiepileptic drugs [8]. In the middle of plant species diversity, the “aromatic plants” have raised interest for their pharmacological and physiological actions, with several properties in the central nervous system (CNS), including antiepileptic activity [9]. These activities have generally been attributed to essential oils and/or their chemical constituents [10], such as phenylpropanoid [11].

*trans*-Anethole (1-methoxy-4-(1-propenyl) benzene) is a phenylpropanoid that is mostly obtained from essential oil of star anise (*Illicium verum*), anise (*Pimpinella anisum*), and sweet fennel (*Foeniculum vulgare*), tarragon (*Artemisia dracunculus L.*) as a major compound [12–14]. *trans*-Anethole (TAN) appears to be responsible for most of essential oil properties attributed to star anise (*Illicium verum*), such as insecticidal [15], antimicrobial and antiviral [16], antioxidant [17], anticarcinogenic [18, 19], anti-inflammatory [20, 21], and antihypernociceptive activities [22]. In tarragon (*Artemisia dracunculus L.*), it is the major substance and the extract has anticonvulsant activity [14]. Thus, isolated TAN has also some properties described as antifungal [23] and anti-inflammatory effects in chronic lung disease [24], but reports of the anticonvulsant activity of this compound isolated are still scarce. So, the activity found in these studies can be attributed, not necessarily to the major compound, but to any of the compounds present in the extract, or even by the association of them. Therefore, we hypothesized that TAN may have an anticonvulsant action as an isolated compound, and to investigate this, we evaluated the effect of TAN in seizure animal models trough behavioral and electroencephalographic methods.

## 2. Material and Methods

### 2.1. Reagents

TAN was obtained from Sigma-Aldrich (Brazil) and solubilized in Tween 80® (5%). Pentylenetetrazole, diazepam, and phenytoin were purchased from Sigma-Aldrich (St. Louis, MO, USA), Hipolabor® (Belo Horizonte, Brazil), and Cristália® (São Paulo, Brazil), respectively, solubilized in saline (NaCl 0.9%) and administered 10 mL/kg of animal.

### 2.2. Animals

Swiss albino male mice (*Mus muscullus L.*), 2-3 months old, weighing 25-35 g were used. The animals were obtained from Professor Thomas George Bioterium of Pharmaceuticals and Medicines Research Institute (IPeFarM)/UFPB. They were housed in polyethylene cages with 4 animals each and maintained under controlled temperature (22 ± 1°C), 55% relative humidity, with a 12 h light/dark cycle (lights on at 6 : 00 a.m.), and food (Purina commercial pellet feed, Paulínia, São Paulo, Brazil) and water available ad libitum. Experimental protocols were performed in accordance with the International Council for Laboratory Animal Science (ICLAS) and were approved by the Ethics Committee on Animal Use/CEUA (certificate no. 3890250918of UFPB).

### 2.3. Experimental Design

Animals were divided randomly into groups and tests were performed between 08:00 and 17:00 h with at least one animal representing each group per day of experiment. All animals were acclimatized 1 h in the laboratory before experiments and 10 minutes inside the experimental box used for electroencephalogram (EEG) record. Each mice was used only once.

### 2.4. Acute Toxicity–LD_50_

TAN acute toxicity study was done according to OECD (Organization for Economic Cooperation and Development) guidelines no.: 423, and low and high doses were selected for treatment. The TAN was administered (i.p.) in escalating dosages, up to 2000 and 1000 mg/kg to different mouse groups (*n* = 3). The animals were observed for behavioral and physiological variations, initially for 4 hours continuously, followed by every 4 and 12 hours and then once a day for fourteen days. If toxic signs or lethality is not observed during the 14 days, the limit test dose is selected for the present investigation.

### 2.5. Maximal Electroshock-Induced Seizure (MES)

Animals were divided into five groups (*n* = 8/group). The vehicle group was treated with saline 0.9% (10 mL/kg, i.p.) and the standard group with phenytoin (25 mg/kg, i.p.) [25]. The experimental groups were treated with different doses of TAN (200, 300, and 400 mg/kg, i.p.). After 30 min of control treatment and 60 min after experimental treatment, seizures were induced by electroshock of 150 pulses/s and 0.5 s duration through auricular clip electrodes (ECT UNIT 7801). The main parameter evaluated was the duration of tonic seizures (complete hind limb extensions) [26].

### 2.6. Pentylenetetrazole-Induced Seizure Test

Anticonvulsant activity evaluation was carried out using PTZ-induced seizure test [27]. Animals were divided into five groups (*n* = 8-10/group). The vehicle control group was treated with saline 0.9% (10 mL/kg, i.p.) and standard group with diazepam (5 mg/kg, i.p.) [28]. The experimental groups were treated with different doses of TAN (200, 300, and 400 mg/kg, i.p.). After 30 min of vehicle treatment and 60 min of experimental treatment, animals were injected with PTZ (75 mg/kg, i.p.). Each animal was observed for latency to first myoclonic jerks, latency to tonic-clonic seizure, seizure duration, and mortality over 15 min [29, 30].

### 2.7. Electrophysiological Study

#### 2.7.1. Stereotaxic Surgery

Animals from PTZ test were submitted previously to a stereotactic surgery to implant electrodes for EEG records during this test. Therefore, animals were anaesthetized with ketamine (70 mg/kg, i.p.) and xylazine (10 mg/kg, i.p.) and placed in a rodent stereotaxic apparatus. Superficially, three stainless steel screw electrodes were placed bilaterally in the parietal cortex. The other one was placed in the frontal cortex as a reference electrode. Electrodes were connected to a multipin socket through welding and fixed to skull with dental acrylic cement. After surgery, animals were treated with central analgesic and antibiotic (i.p.). All experiments were performed 4–5 days after stereotaxic surgery.

#### 2.7.2. EEG Recordings: PTZ Test

Before PTZ experiment, surgical animals were brought to a laboratory to acclimatize. Animals were connected to a digital encephalograph equipment (Neuromap EQSA260, Neuromap LTDA, Brazil) through an electrode preinstalled in stereotaxic surgery and put into a glass box, one per time, to register the electrophysiological brain activity during the experiment. To establish an adequate control period, EEG signals were recorded for 10 minutes before substance administration, as a baseline, 60 minutes following treatments, and 15 minutes after PTZ administration. The EEG signals were filtered (0.1 to 60.0 Hz, bandpass), stored in a computer, and analyzed later using LabChart 7.0 software (AD instruments). Wave amplitudes were automatically calculated using average cyclic height by LabChart function. Analysis of this experiment was done in order to obtain the most reliable data as possible. Therefore, the middle session of basal and treatment EEG was analyzed, and to analyze seizures induction, initial data after PTZ administration was analyzed.  Figure 1 shows the experimental design of the pentylenetetrazole (PTZ) test accompanied by EEG and design of vehicle and diazepam administration.

### 2.8. Statistical Analysis

The normality of data was made by Shapiro-Wilk test and Brown Forsythe test was applied to verify variance homogeneity. The behavioral data was analyzed by one-way analysis of variance (ANOVA). Tukey test was applied in parametric data (MES) for multiple comparisons between groups' mean and the mean of vehicle group. Data was represented as mean ± standard deviation. Behavioral data for seizures induced by PTZ is nonparametric and therefore were analyzed by Kruskal-Wallis test followed by Dunn's post hoc when appropriate for multiple comparisons between groups' mean and the mean of vehicle group. Data were presented as median and interquartile ranges. EEG analysis were done by two-way ANOVA followed by Tukey test for multiple comparisons between groups' mean and the mean of vehicle group. Data was represented as mean ± standard error of the mean. Mortality percentage was calculated using Fisher's exact test. *H* values were considered significant and presented only when *p* < 0.05.

## 3. Results

### 3.1. Acute Toxicity Study

In acute toxicity test, TAN 2000 mg/kg (i.p.) caused animal group mortality in less than 48 hours. The experiment was repeated with TAN at 1000 mg/kg (i.p.) dose, and there was no sign of acute toxicity or animal death in this group during the 14 days of observation. Therefore, the LD50 was estimated in 1000 mg/kg.

### 3.2. Maximal Electroshock-Induced Seizure (MES)

The tonic seizure duration in MES test was decreased in TAN 300 mg/kg (12.00 ± 2.9 s) and 400 mg/kg (9.00 ± 4.4 s) groups compared to vehicle (21.71 ± 6.5 s). The phenytoin group (2.29 ± 1.7 s) as predicted was able to significantly attenuate electrically induced seizures (*F* (4.35) = 26.21), as observed in Figure 2.

### 3.3. Pentylenetetrazole-Induced Seizure Test

The effect of TAN in PTZ-induced seizures is shown in Figure 3. TAN at 400 mg/kg (80.0 (56.0–134.0)) statistically increased latency for the first myoclonic jerk (*p* < 0.05), as did DZP (5 mg/kg) (144.0 (76.0–900)), *p* < 0.0001, compared to vehicle (control group) (34.0 (10.0–82.0); *H* (4) = 23.17) (Figure 3(a)). TAN 400 mg/kg (900.0 (861.0–900.0)) increased latency to tonic-clonic seizure as shown in Figure 3(b), demonstrating a similar result as the DZP group (5 mg/kg) (900.0 (900.0–900.0)) compared to vehicle (90.0 (23.0–160.0); *H* (4) = 33.3; *p* < 0.0001).

As for the parameter duration of tonic-clonic seizures, just TAN 400 mg/kg (0.0 (0.0–10.0)) and diazepam (0.0 (0.0–16.0)) were able to decrease seizure duration compared to the vehicle group (20 (8–52.0); *H* (4) = 28.97; *p* < 0.0001) (Figure 3(c)). The animals treated with TAN at 300 and 200 mg/kg doses did not express significantly results in those parameters mentioned above.

Moreover, no animal deaths in TAN (400, 300, and 200 mg/kg) and DZP pretreated groups were observed. The same could not be applied to the vehicle group that showed 75% of group mortality (Table 1).

### 3.4. Electroencephalogram Registers

The quantitative results presented in Figure 3 are corroborated by the EEG recording data exposed in Figure 4. These graphics show EEG amplitude register data over experiment time, in which *a* and *b* represent 3 minutes of the middle section of baseline and treatment, respectively, and *c* is the initial 3 minutes right after PTZ injection. In baseline, there was no significantly difference between groups (a), while animals treated with TAN had an amplitude decrease compared to control groups in treatment section (b) (*F* (4, 37) = 22.1, *p* < 0.0001). After 1 minute of PTZ injection, TAN 300, TAN 400, and DZP groups significantly decreased wave amplitude compared to control (c) (*F* (4, 37) = 10.26, *p* < 0.0001).

Figures 4(d)–4(f) shows the same result described before, calculated as mean of total amplitude, instead. The average of the same period shows that TAN 400 mg/kg (1.06 ± 0.16), 300 mg/kg (1.82 ± 0.23) and standard diazepam group (0.90 ± 0.06) (*F* (4, 40) = 13.01, *p* < 0.0001) demonstrated a reduction in the amplitude compared to the vehicle group (2.48 ± 0.12).

Each group represented in Figure 4(c) was separated for better visualization with their respective EEG record representation beside (Figures 5(a)–5(j)). In this figure, it is possible to observe a wave amplitude decrease of TAN 200, 300, and 400 and DZP groups compared to vehicle (PTZ). EEG records also show that TAN 300 (Figures 5(e) and 5(f)) and 400 (Figures 5(g) and 5(h)) were able to increase the latency to myoclonic jerk appearance, attenuating/inhibiting generalized tonic-clonic seizures as presented in behavioral previews results.

## 4. Discussion

This study showed that TAN acute intraperitoneal administration has antiseizure potential in behavioral and electroencephalographic studies. This substance was able to inhibit and/or attenuate seizures in MES and PTZ models in mice, and no death was verified on experimental groups.

Since ancient times, innumerous aromatic species had been employed for their medicinal properties. A review study reported that some plant species possess essential oils compounds with anticonvulsant activity in experimental models of seizure [9, 10]. They show many pharmacological effects on CNS, including anticonvulsant activity, and it is probably due to the high structural diversity of constituents, like the monoterpene epoxy-carvone [30], terpinen-4-ol [31], alpha and beta-pinene [32], and the phenylpropanoid eugenol [11]. TAN is a phenylpropanoid, obtained, principally, from the essential oil of star anise (*Illicium verum*), as a majority component [15, 23]. In this work, acute toxicity tests according to OECD 423 demonstrated that TAN LD_50_ was estimated at 1.000 mg/kg and no death or toxic signs were observed during 14 days; therefore, doses were chosen about one third of this value for the experiments.

In the attempt to find a natural compound for an adequate epilepsy treatment, this study was carried out to evaluate whether TAN exhibits effects in MES and/or PTZ seizure models. Investigating TAN action in MES test, it was observed that 300 and 400 mg/kg doses were able to reduce tonic seizures duration compared to the vehicle group, in a similar way to the standard drug used (phenytoin). MES test is a consolidated model and widely used in screenings for anticonvulsant agent development [33]. It is based on electrical discharges application for a short period of time, leading to depolarization of sodium channels causing neuron excitability that can trigger seizures [34]. Like TAN in this work, drugs as phenytoin and lamotrigine that inhibit voltage-dependent Na^+^ channels and attenuate MES-induced tonic seizures have potential to prevent electrical discharge spread through neurons, decreasing seizures duration and increasing threshold for new crises appearance, therefore being characterized as potential anticonvulsant agents [35, 36].

It has been described that many essential oils and its compounds have anticonvulsant activity in animal models as MES and PTZ tests [33]. A study demonstrated that the essential oil of *Thymus vulgaris* promotes protection against MES-induced seizures. The essential oil in a fixed dose of 300 mg/kg, a similar dose used in the present study by the same intraperitoneal route, also showed greater protection against convulsions induced by electrical discharges [37]. Among the main compounds isolated from this oil, there are borneol and thymol. Interestingly, both compounds were found to have a highly positive modulating action at GABA_A_ receptors [38, 39]. In this way, electrical discharges may be contained by the increasing action of GABAergic pathway that inhibits neuronal transmission.

Pentylenetetrazole-induced seizure test is another standard method of anticonvulsant screening [40]. PTZ promotes seizures inhibiting GABA activity at GABA_A_ receptors causing an excitation/inhibition imbalance mechanism leading to neuronal hyperexcitability [41]. Drugs that attenuates seizures or increases latency to first myoclonic jerk and/or to tonic-clonic seizures in PTZ test are considerate anticonvulsant agents [42]. Benzodiazepines, like diazepam, is expected to block seizures, due to its ability to open GABA_A_ channels and facilitating GABAergic transmission [43].

In this test, TAN highest dose (400 mg/kg) increased latency to myoclonic jerks and tonic-clonic seizure compared to the vehicle group, as reduced the duration of generalized seizures. TAN showed a similarly result compared to animals treated with DZP, a standard drug used in the clinic, demonstrating a protective effect. The fact that TAN inhibits PTZ-induced seizures may be indicative of its involvement in GABAergic transmission. However, more experiments need to be done. A related study with isopentyl ferulate, a compound belonging to the same class as the TAN phenylpropanoid, demonstrated anticonvulsant activity against PTZ-induced seizures at 25, 50, and 75 mg/kg doses. The researchers showed that a pretreatment with flumazenil, a GABA receptor antagonist, reversed the anticonvulsant action of isopentyl ferulate, indicating GABAergic modulation. When compared with this study, the compound isopentyl ferulate demonstrated anticonvulsant action, but it was not able to protect the animals against death. Data showed 50-75 percentage of the animal deaths, while TAN protection was extended to animal mortality rate and there were no deaths in TAN-treated groups [44].

We also investigated the TAN electroencephalography profile. During this substance treatment, animals had an amplitude of wave decrease compared to vehicle and DZP groups, indicating CNS depressant activity. EEG data also corroborates with behavioral findings, once TAN attenuates behavioral and EEG alterations induced by PTZ. This can be observed due to PTZ ability to increase spikes appearance and neuronal firing rate frequency, being an indicator of neuronal excitability increase commonly observed in seizure processes [45]. TAN-treated groups presented less EEG alterations and amplitude quantification shows that TAN 300 and 400 mg/kg doses were able to prevent amplitude increase induced by PTZ, as did DZP treatment, demonstrating an antiseizure effect. A decrease in the number of spikes can also be observed, as well as an increase to the onset time to spikes appearance right after PTZ administration. This indicated reduction of paroxystic activity severity that was confirmed by behavioral symptoms [31].

The attenuation of convulsions in MES, PTZ-induced seizure tests, and EEG results by TAN pretreatment suggests its direct or indirect effect on brain excitatory/inhibitory mechanisms in accordance to Boissier classic study [46]. In line with these findings, it has been demonstrated that TAN can modify the function of Ca^2+^ channels and K^+^-activated Ca^2+^ channels, which may be involved with changes in brain cell membrane potential and the consequent neurotransmission [47]. In addition, TAN seems to act in other channels, like the receptor GABA_A_, to attenuate seizures in the MES test. As other essential oil compounds like borneol [38] and thymol [39], TAN seems to enhance the GABAergic pathway preventing the propagation of neuronal firings caused by electrical discharges. This hypothesize can be corroborated by the fact that TAN also possess anticonvulsant activity against PTZ-induced seizures, similarly to the isopentyl ferulate, a compound that belongs to the same class of phenylpropanoids. Once PTZ mechanisms of action involves the GABA pathway block, the reversal of seizure induced by this substance is indicative of via GABAergicaction; however, further studies on the mechanism of action need to be carried out [44].

In addition, the presence of TAN prevented excitotoxicity induced by the addition of NMDA in an in vitro model of cerebral ischemia, demonstrating that it can act on the functioning of glutamatergic receptors [48]. Meanwhile, a study carried out molecular docking analysis [49] suggest *β*3-adrenergic receptor as a possible target of action of TAN, and since these receptors are expressed in several brain areas [50], we can presuppose that this is another way in which the substance acts causing an antidepressant effect in mice [51], as well as the antiseizure effect seen in our study.

Moreover, TAN appears to be responsible for the properties attributed to essential oil of *Illicium verum*, such as antioxidant activities [17]. Studies have shown that anethole antioxidant effect is attributable to its ability to sequester free radicals, decreasing reactive oxygen species concentrations [20, 52]. Its antioxidant activity is similar to other phenolic compounds, being dependent on conjugated double bonds [20]. Thus, anethole can increase intracellular levels of glutathione and glutathione-S-transferase, inhibiting lipid peroxidation [20, 53]. Glutathione is an endogenous antioxidant form within free radicals and prevents hydroxyl radical generation, the most toxic form of free radicals [54]. In this context, TAN might be able to attenuate seizures and free radical-induced neurodegeneration, but more detailed pharmacological studies are needed to better elucidate what are the multiple mechanisms involved in antiseizure and neuroprotective activities of TAN.

Finally, our results emphasize the importance of new pharmacotherapeutic alternative research, through the infinite arsenal of natural resources available. Given its extreme reach, this is a challenging area, but still offers a vast field for new drug discovery and development.

## 5. Conclusion

*trans*-Anethole demonstrated potential antiseizure properties in behavioral and encephalographic studies. TAN 400 mg/kg dose showed the best effect being able to decrease the duration of tonic seizures in MES and tonic-clonic seizures in PTZ-induced models in mice. Furthermore, this dose increases the onset time to the first myoclonic jerk and tonic-clonic seizure appearance, protecting animals from death in the PTZ test. Also, the EEG profile revealed that TAN inhibit and/or attenuate seizures reducing amplitude of brain waves.

However, further research still needed to be carried on these and other animal models, using pharmacological tools and neurochemical analyzes for a better understanding of the mechanism of action by which TAN alters EEG records, protects against induced seizures, and has a probable neuroprotective effect. This clarification is extremely important before testing this substance as a therapeutic alternative for the treatment of epilepsy in humans.

## Figures and Tables

**Figure 1:** Experimental design of the pentylenetetrazole (PTZ) test accompanied by EEG. Design of vehicle and diazepam administration (a) and *trans*-anethole (TAN) groups (b). Arrows indicate substance administration.

**Figure 2:** Effect of *trans*-anethole in duration of tonic seizures induced by maximum electroshock in seconds. Groups: vehicle (Tween 80, 5%), *trans*-anethole (TAN; 200, 300, and 400 mg/kg), and phenytoin (25 mg/kg). Analysis of data by one-way ANOVA, followed by the Tukey test. ^∗∗∗^*p* < 0.001 and ^∗∗∗∗^*p* < 0.0001 compared to the vehicle (control). The values represent the mean ± standard deviation (*n* = 8 group/group).

**Figure 3:** Effect of *trans*-anethole in PTZ-induced seizures (PTZ, 75 mg/kg; i.p.). Vehicle (5% tween 80), *trans*-anethole (TAN; 200, 300, and 400 mg/kg), and diazepam (DZP; 5 mg/kg) groups. (a) Latency to myoclonic jerks, (b) latency to tonic-clonic seizure, and (c) duration of tonic-clonic seizure results after PTZ injection in seconds. Values represent the median and interquartile ranges compared to vehicle (*n* = 8-10/group). The data were analyzed by one-way ANOVA, followed by the Kruskal-Wallis test and post hoc Dunn's, ^∗∗∗^*p* < 0.001 and ^∗∗∗∗^*p* < 0.0001.

**Figure 4:** Effect of TAN (200, 300, or 400 mg/kg, i.p.) administration on EEG recording after pentylenetetrazole-induced seizure test. The data were normalized by the average of the total baseline period (10 minutes) and presented as the average (line) of every 20 seconds of (a) amplitude of baseline, 3 minutes of middle section; (b) amplitude of treatment, 3 minutes of middle section; and (c) amplitude of initial 3 minutes after PTZ injection. Bar graphics represent the same data analyzed as total mean of (d) amplitude of baseline, 3 minutes of middle section; (e) amplitude of treatment, 3 minutes of middle section; and (f) amplitude of initial 3 minutes section after PTZ injection. Values represent the mean ± standard error of the mean (*n* = 6–10/group). Two-way ANOVA followed by Tukey test. “*a*” indicates a difference between the DZP and TAN 400 mg/kg groups compared to vehicle; “*b*” indicates a difference between TAN 300 mg/kg and vehicle; and “*c*” differentiates TAN groups compared to vehicle and DZP. ^∗∗^*p* < 0.01, ^∗∗∗∗^*p* < 0.0001 compared to the vehicle group.

**Figure 5:** Quantification of amplitude (derived from Figure 4(c) (*n* = 6-10/group) and the, respectively, representative electroencephalographic record (EEG) beside. Graphs represent one animal of each group (randomly chosen) after pentylenetetrazole (PTZ; 75 mg/kg, ip) injection. Groups: vehicle (5% Tween 80) (a, b), *trans*-anethole: TAN 200 mg/kg (c, d), TAN 300 mg/kg (e, f), TAN 400 mg/kg (g, h), and diazepam: DZP 5 mg/kg (i, j). The arrow indicates first alteration on EEG induced by PTZ.

**Table 1:** *trans*-Anethole (TAN) and diazepam (DZP) effects on mortality percentage during 15 minutes after PTZ-induced seizure test. Fisher's exact test, ^∗∗∗^*p* < 0.001; compared to the vehicle group (*n* = 8-10/group).

Groups	Dose	Mortality (%)
Vehicle	___	75

*trans*-Anethole	200 mg/kg	0^∗∗∗^
	300 mg/kg	0^∗∗∗^
	400 mg/kg	0^∗∗∗^

Diazepam	5 mg/kg	0^∗∗∗^

## Data Availability

All related data are in the manuscript.
